# A Method for Detecting Incipient Faults in Satellites Based on Dynamic Linear Discriminant Analysis

**DOI:** 10.1155/2021/1303936

**Published:** 2021-10-14

**Authors:** Ge Zhang, Qiong Yang, Guotong Li, Jiaxing Leng

**Affiliations:** ^1^Innovation Academy for Microsatellites of CAS, Shanghai 201203, China; ^2^University of Chinese Academy of Sciences, Beijing 100049, China; ^3^School of Information Science and Technology, ShanghaiTech University, Shanghai 201210, China

## Abstract

Timely detection and treatment of possible incipient faults in satellites will effectively reduce the damage and harm they could cause. Although much work has been done concerning fault detection problems, the related questions about satellite incipient faults are little addressed. In this paper, a new satellite incipient fault detection method was proposed by combining the ideas of deviation in unsupervised fault detection methods and classification in supervised fault detection methods. First, the proposed method uses dynamic linear discriminant analysis (LDA) to find an optimal projection vector that separates the in-orbit data from the normal historical data as much as possible. Second, under the assumption that the parameters obey a multidimensional Gaussian distribution, it applies the normal historical data and the optimal projection vector to build a normal model. Finally, it employs the noncentral *F*-distribution to test whether a fault has occurred. The proposed method was validated using a numerical simulation case and a real satellite fault case. The results show that the method proposed in this paper is more effective at detecting incipient faults than traditional methods.

## 1. Introduction

With the reduction in the costs of launching rockets and manufacturing satellites, the number of satellites operating in orbit increases annually, bringing large economic benefits to society [1–3]. However, due to the harsh operating environment of satellites and human error, key modules or components of satellites in orbit may have abnormalities or experience failures [4]. If incipient faults can be detected and dealt with promptly in their early stages, the damage and harm they cause will be effectively reduced [5]. Therefore, the detection of incipient faults in satellites is receiving an increasing amount of attention because it is one of the key technologies that ensures the normal operation of satellites [6, 7].

The current common method used to detect faults in satellites is to compare telemetry parameters with preset thresholds directly [8, 9]. This fault detection method is suitable for detecting abrupt and large faults. However, it may be less effective at detecting incipient faults because the telemetry parameters with an incipient fault may not change significantly from their normal condition [10]. If the fault detection threshold was set too low, the fault detection method would be sensitive to noise and cause frequent false alarms; whereas if the threshold was set too high, some early symptoms of the fault might be missed. In addition, as the production batches, processes, and operating environments of different satellites are not identical, different fault detection thresholds may need to be determined for different satellites, and it is inefficient to manually set the appropriate threshold for each telemetry parameter.

Model-based satellite fault detection methods are more intelligent than threshold comparison methods and often combine fault detection, isolation, and recovery functions [11–13]. However, with the rapid development of science and technology, a variety of new technologies, materials, and highly integrated devices are being used in satellites. The complex coupling relationships between the various components of a satellite and the lack of familiarity of various faults can make it difficult to build accurate and comprehensive fault detection models, thus limiting the application of model-based satellite fault detection methods.

In recent years, data-driven fault detection methods have become a popular research topic due to the advantages of low expert involvement, high modeling efficiency, and high scalability [14–16]. At present, data-driven fault detection methods are mainly divided into two categories: unsupervised fault detection methods and supervised fault detection methods. The core idea of unsupervised fault detection methods is deviation. These methods use the normal historical data to automatically build a model that characterizes the normal condition of the satellite. It assumes that a fault has occurred when the actual in-orbit data deviates significantly from the model characterizing the normal data. Since the ground test data and the in-orbit data of satellites contain mostly fault-free data, fault detection methods based on unsupervised learning have been widely researched and applied. Representative unsupervised fault detection methods are one-class support vector machine (OCSVM) [17], inductive monitoring system (IMS) [18], principal component analysis (PCA) [19], Gaussian process regression (GPR) [20], long short-term memory (LSTM) [21], and so on. Although these methods use different principles to build normal models, they all have one thing in common—all normal models used to detect faults are obtained by learning from the normal historical data. Once the learning process is complete, each method will use a fixed and invariable model to detect faults, regardless of the variation of the actual in-orbit data, with no optimization or adjustment for the actual faults that may occur.

The core idea of supervised fault detection methods is classification. These methods learn and build a classifier from the normal historical data and various real or simulated fault data. If the in-orbit data were classified as a normal class by the classifier, the in-orbit data would be free of faults. Conversely, if the in-orbit data were classified as a fault class by the classifier, the in-orbit data would be deemed to be faulty in some way. Representative supervised fault detection methods are linear discriminant analysis (LDA) [22], support vector machine (SVM) [23], neural networks [24], random forest [25], and so on. However, due to the high reliability of satellites, most of the samples collected by satellite operation and maintenance systems are normal, and fault samples are exceedingly rare. In addition, the classification models built using the fault samples from different satellites may not be generalized, thus hindering the application of supervised fault detection methods in the satellite domain.

Based on the existing research, this paper proposes a new satellite incipient fault detection method that combines the ideas of deviation in unsupervised fault detection methods and classification in supervised fault detection methods. The main contributions of our work are summarized as follows:

1. This paper first uses the idea of classification to find an optimal projection vector separating the in-orbit data from the normal historical data. Specifically, this paper considers the fault detection problem as a binary classification problem and uses LDA to find the optimal projection vector where the in-orbit telemetry data can be distinguished from the normal historical data to the greatest extent.
2. This paper then uses the idea of deviation to test whether a fault has occurred in the in-orbit data. Specifically, a normal model is built using the normal historical data and the optimal projection vector, and the fault is determined by testing whether the deviation of the in-orbit data from the normal model exceeds the threshold.

This paper is organized as follows: A brief introduction about LDA is given in Section 2. The fault detection method based on dynamic LDA is presented in detail in Section 3. Then, the proposed method is illustrated and analysed using a numerical simulation case and a real satellite fault case in Section 4. Finally, conclusions are given in Section 5.

## 2. Linear Discriminant Analysis

Linear discriminant analysis, also known as Fisher discriminant analysis [26], is a supervised dimensionality reduction and classification method which is widely used in the field of pattern recognition and machine learning [27–29]. Taking the binary classification as an example, given a data set *D*={(*x*_*i*_, *z*_*i*_)}_*i*=1_^*n*^, where *x*_*i*_ ∈ *R*^*m*^ is a column vector of multidimensional telemetry parameters, *z*_*i*_ ∈ *R* is the corresponding class label, *m* is the number of variables need be monitored, and *n* is the is the number of samples. There are only two values of *z*_*i*_, *z*_*i*_ ∈ {0,1}. Let *n*_*j*_ ∈ *R*, *X*_*j*_ ∈ *R*^*n*_*j*_×*m*^, *μ*_*j*_ ∈ *R*^*m*^, and Σ_*j*_ ∈ *R*^*m*×*m*^, respectively, represent the number of samples, the set of samples, the mean vector, and the covariance matrix of the class *j*, *j* ∈ {0,1}.

We assume that the projection vector is *w* ∈ *R*^*m*^. For each sample *x*_*i*_, the projection of *x*_*i*_ onto the vector *w* is *w*^*T*^*x*_*i*_. Moreover, the projections of *μ*_0_ and *μ*_1_ onto the vector *w* are *w*^*T*^*μ*_0_ and *w*^*T*^*μ*_1_, respectively. The scatter of each class after projection onto the vector *w* is *S*_*j*_^2^, as shown in

(1) $$\begin{array}{c} S_{j}^{2}=\sum_{x\in X_{j}}{\left(w^{T}x-w^{T}\mu_{j}\right)}^{2},\;j\in \left\{0,1\right\}. \end{array}$$

We expect that the samples of the same class are clustered together as much as possible after projection onto the vector *w*, while the samples of different classes to be more dispersed [30]. Thus, we can construct the objective function of LDA *J*(*w*), as shown in

(2) $$\begin{array}{c} J\left(w\right)=\frac{{\left\|w^{T}\mu_{0}-w^{T}\mu_{1}\right\|}_{2}^{2}}{S_{1}^{2}+S_{2}^{2}}=\frac{w^{T}S_{b}w}{w^{T}S_{w}w}. \end{array}$$

In equation (2), *S*_*b*_=(*μ*_0_ − *μ*_1_)(*μ*_0_ − *μ*_1_)^*T*^ and *S*_*w*_=Σ_0_+Σ_1_. The objective of LDA is to find an optimal projection vector *w* that maximizes *J*(*w*). Let *w*^*T*^*S*_*b*_*w*=1, the problem of finding the optimal projection vector *w* can be transformed into an optimization problem, as shown in

(3) $$\begin{array}{c} \left\{\begin{array}{cc} \max & w^{T}S_{b}w,\\ \text{s.t.} & w^{T}S_{w}w=1. \end{array}\right. \end{array}$$

The optimization problem in equation (3) can be solved by Lagrange multiplier method and then we obtain

(4) $$\begin{array}{c} S_{w}^{-1}S_{b}w=\lambda w. \end{array}$$

From equation (4) and the relationship between eigenvalues and eigenvectors [30], we can know that the projection vector *w* is an eigenvector of the matrix *S*_*w*_^−1^*S*_*b*_. Furthermore, the optimal projection vector *w* is the eigenvector corresponding to the largest eigenvalue of the matrix *S*_*w*_^−1^*S*_*b*_.

## 3. Incipient Fault Detection Method Based on Dynamic LDA

### 3.1. Dynamic LDA

The training data of traditional LDA contain both normal (class 0) and fault (class 1) samples. However, in the field of satellite fault detection, majority of samples available for training are normal samples. Therefore, this paper proposes a new method that treats the normal historical samples as normal (class 0) samples and treats the in-orbit samples which need to be tested as fault (class 1) samples. The traditional use of LDA and the new use of LDA in this paper are shown in Figures 1(a) and 1(b), respectively.

This article intends to use sliding windows and hypothesis testing methods to test whether a fault has occurred in the in-orbit data. The general idea of fault detection is as follows:

1. Sliding windows with the length of *n*_1_ are used to extract the in-orbit data in real time. Let the in-orbit data in the *k*th sliding window be *X*_*k*_ ∈ *R*^*n*_1_×*m*^. We assume that a fault has occurred in *X*_*k*_, and *X*_*k*_ belongs to a different class from the normal historical data *X*_0_ ∈ *R*^*n*_0_×*m*^.
2. LDA is used to find an optimal projection vector *w*_*k*_ ∈ *R* that separates the normal historical data *X*_0_ from the in-orbit fault data *X*_*k*_ as much as possible.
3. A normal model is built using the normal historical data *X*_0_ and the optimal projection vector *w*_*k*_.
4. Whether the in-orbit data *X*_*k*_ deviates significantly from the normal model is tested. If there was a significant deviation, then the original hypothesis that *X*_*k*_ and *X*_0_ belong to different classes is valid, and a fault has occurred in *X*_*k*_. If there was no significant deviation, then the original hypothesis is not valid, and there is no fault in *X*_*k*_.

As can be seen earlier, the traditional use of LDA is static. The optimal projection vector will be fixed once the training data are determined. The new use of LDA in this paper is dynamic. For each sliding window of the in-orbit data *X*_*k*_, an optimal projection vector *w*_*k*_ is obtained using dynamic LDA. As the in-orbit data *X*_*k*_ may vary from different windows, the optimal projection vector *w*_*k*_ may not be the same for each LDA process. Due to the use of dynamic LDA, the optimal projection vectors can adjust the in-orbit data in real time, making the proposed method more adaptable to potential faults.

### 3.2. Construction of the Normal Model

After the optimal projection vector *w*_*k*_ is obtained, we need to verify whether there is a significant deviation between *X*_*k*_ and *X*_0_. However, how large of the deviation is the significant deviation? Therefore, we need to determine the normal fluctuation range of deviation between *X*_*k*_ and *X*_0_ when the in-orbit data *X*_*k*_ is normal, and then use the normal fluctuation range to build a normal model. A fault is considered to have occurred when the deviation is outside the acceptable range.

In this paper, the objective function of LDA *J*(*w*) is used as the measure of deviation. We assume that the normal historical data *X*_0_ ∈ *R*^*n*_0_×*m*^ and the in-orbit data *X*_*k*_ ∈ *R*^*n*_1_×*m*^ obey two *m*-dimensional joint Gaussian distributions *X*_0_ ~ *ℕ*(*μ*_0_, Σ_0_) and *X*_*k*_ ~ *ℕ*(*μ*_*k*_, Σ_*k*_), respectively. The projections of *X*_0_ and *X*_*k*_ onto the vector *w*_*k*_ are *f* ∈ *R*^*n*_0_^ and *g* ∈ *R*^*n*_1_^, respectively. Based on the property of the *m*-dimensional joint Gaussian distribution [31], it is clear that *f* and *g* obey one-dimensional Gaussian distributions *f* ~ *ℕ*(*w*_*k*_^*T*^*μ*_0_, *w*_*k*_^*T*^Σ_0_*w*_*k*_) and *g* ~ *ℕ*(*w*_*k*_^*T*^*μ*_*k*_, *w*_*k*_^*T*^Σ_*k*_*w*_*k*_), respectively. The relationship of *J*(*w*_*k*_), *f*, and *g* is shown in

(5) $$\begin{array}{c} J\left(w_{k}\right)=\frac{{\left\|w_{k}^{T}\mu_{0}-w_{k}^{T}\mu_{k}\right\|}_{2}^{2}}{w_{k}^{T}\left(\Sigma_{0}+\Sigma_{k}\right)w_{k}}. \end{array}$$

Since *X*_0_ and *w*_*k*_ have been obtained after using LDA, it can be considered that the mean vector *μ*_0_, the covariance matrix Σ_0_, and the optimal projection vector *w*_*k*_ in equation (5) are known and fixed, while the mean vector *μ*_*k*_ and covariance matrix Σ_*k*_ associated with *X*_*k*_ are unknown and variable. As *μ*_0_, Σ_0_, and *w*_*k*_ are all known, we can assume that *w*_*k*_^*T*^*μ*_0_=*c*_1_ and *w*_*k*_^*T*^Σ_0_*w*_*k*_=*c*_2_, where *c*_1_ and *c*_2_ are two constants. Then, equation (5) can be reduced to

(6) $$\begin{array}{c} J\left(w_{k}\right)=\frac{G_{1}\left(w_{k}\right)}{G_{2}\left(w_{k}\right)}=\frac{{\left\|w_{k}^{T}\mu_{k}-c_{1}\right\|}_{2}^{2}}{c_{2}+w_{k}^{T}\Sigma_{k}w_{k}}. \end{array}$$

For the purpose of obtaining the normal fluctuation range of *J*(*w*_*k*_), we assume that *X*_*k*_ and *X*_0_ belong to the same class and *X*_*k*_ is obtained by sampling the joint Gaussian distribution which *X*_0_ obeys. Since *f* and *g* obey one-dimensional Gaussian distributions and are the projections of *X*_*k*_ and *X*_0_ onto the vector *w*_*k*_, respectively, we can consider that *g* is obtained by sampling the one-dimensional Gaussian distribution which *f* obeys. Based on the property of the one-dimensional Gaussian distribution [32, 33], the sample mean value *w*_*k*_^*T*^*μ*_*k*_ of *g* obeys a one-dimensional Gaussian distribution, as shown in equation (7). (*n*_1_ − 1)*w*_*k*_^*T*^Σ_*k*_*w*_*k*_/*w*_*k*_^*T*^Σ_0_*w*_*k*_ obeys the chi-square distribution with degrees of freedom of *n*_1_ − 1 [32, 33], as shown in the following equations:

(7) $$\begin{array}{c} w_{k}^{T}\mu_{k}∼\mathbb{N}\left(w_{k}^{T}\mu_{0},\frac{w_{k}^{T}\Sigma_{0}w_{k}}{n_{1}}\right), \end{array}$$

(8) $$\begin{array}{c} \frac{\left(n_{1}-1\right)w_{k}^{T}\Sigma_{k}w_{k}}{w_{k}^{T}\Sigma_{0}w_{k}}∼\chi^{2}\left(n_{1}-1\right). \end{array}$$

Since *w*_*k*_^*T*^*μ*_*k*_ obeys a one-dimensional Gaussian distribution and *c*_1_ is a constant, *w*_*k*_^*T*^*μ*_*k*_ − *c*_1_ also obeys a one-dimensional normal distribution, as shown in

(9) $$\begin{array}{c} w_{k}^{T}\mu_{k}-c_{1}∼\mathbb{N}\left(w_{k}^{T}\mu_{0}-c_{1},\frac{w_{k}^{T}\Sigma_{0}w_{k}}{n_{1}}\right). \end{array}$$

As *w*_*k*_^*T*^*μ*_0_=*c*_1_ and *w*_*k*_^*T*^Σ_0_*w*_*k*_=*c*_2_, we can obtain

(10) $$\begin{array}{c} w_{k}^{T}\mu_{k}-c_{1}∼\mathbb{N}\left(0,\frac{c_{2}}{n_{1}}\right). \end{array}$$

After normalizing *w*_*k*_^*T*^*μ*_*k*_ − *c*_1_, we can obtain

(11) $$\begin{array}{c} \sqrt{\frac{n_{1}}{c_{2}}}\left(w_{k}^{T}\mu_{k}-c_{1}\right)∼\mathbb{N}\left(0,1\right). \end{array}$$

Furthermore, we can get equation (12) from the relationship between the standard normal distribution and the chi-square distribution:

(12) $$\begin{array}{c} \frac{n_{1}}{c_{2}}{\left\|w_{k}^{T}\mu_{k}-c_{1}\right\|}_{2}^{2}∼\chi^{2}\left(1\right). \end{array}$$

Thus, the numerator of *J*(*w*_*k*_) satisfies

(13) $$\begin{array}{c} \frac{n_{1}}{c_{2}}G_{1}\left(w_{k}\right)∼\chi^{2}\left(1\right). \end{array}$$

Using *w*_*k*_^*T*^Σ_0_*w*_*k*_=*c*_2_ to simplify equation (8), we can get

(14) $$\begin{array}{c} \frac{\left(n_{1}-1\right)w_{k}^{T}\Sigma_{k}w_{k}}{c_{2}}∼\chi^{2}\left(n_{1}-1\right). \end{array}$$

Therefore, the denominator of *J*(*w*_*k*_) satisfies

(15) $$\begin{array}{c} \frac{\left(n_{1}-1\right)}{c_{2}}\left(G_{2}\left(w_{k}\right)-c_{2}\right)∼\chi^{2}\left(n_{1}-1\right). \end{array}$$

In summary, the numerator of *J*(*w*_*k*_) multiplied by a constant *n*_1_/*c*_2_ obeys a chi-square distribution with a 1 degree of freedom. The denominator of *J*(*w*_*k*_) minus a constant *c*_2_ and then multiplied by a constant (*n*_1_ − 1)/*c*_2_ obeys a chi-square distribution with *n*_1_ − 1 degrees of freedom. Therefore, the denominator of *J*(*w*_*k*_) obeys a noncentral chi-square distribution. In addition, *G*_1_(*w*_*k*_) and *G*_2_(*w*_*k*_) are independent of each other. The relationship between the chi-square distribution and the *F*-distribution and equations (13), (15) show that 1/*n*_1_*J*(*w*_*k*_) obeys a noncentral *F*-distribution with degrees of freedom of *n*_1_ − 1 and 1 and a noncentral parameter *c*_2_, as shown in

(16) $$\begin{array}{c} \frac{1}{n_{1}J\left(w_{k}\right)}=\frac{G_{2}\left(w_{k}\right)}{n_{1}G_{1}\left(w_{k}\right)}=\frac{n_{1}-1/c_{2}*G_{2}\left(w_{k}\right)/n_{1}-1}{n_{1}/c_{2}*G_{1}\left(w_{k}\right)/1}∼F\left(n_{1}-1,1,c_{2}\right). \end{array}$$

Therefore, we can use the noncentral *F*-distribution to test whether there is a fault in *X*_*k*_ [33]. Given a significance level *α*, the detection threshold *ε*_*k*_ ∈ *R* of 1/*n*_1_*J*(*w*_*k*_) can be obtained from the noncentral *F*-distribution test. If the value of 1/*n*_1_*J*(*w*_*k*_) was greater than or equal to *ε*_*k*_, we consider that *X*_*k*_ and *X*_0_ belong to the same class, and there is no fault in *X*_*k*_. If the value of 1/*n*_1_*J*(*w*_*k*_) was less than *ε*_k_, we consider that *X*_*k*_ and *X*_0_ belong to different classes and a fault has occurred in *X*_*k*_. Taking the reciprocal of 1/*n*_1_*J*(*w*_*k*_), we can obtain

(17) $$\begin{array}{c} \left\{\begin{array}{c} H_{0}:J\left(w_{k}\right)\leq \frac{1}{n_{1}\varepsilon_{k}},\;\text{fault}-\text{free,}\\ H_{1}:J\left(w_{k}\right)>\frac{1}{n_{1}\varepsilon_{k}},\;\text{faulty.} \end{array}\right. \end{array}$$

### 3.3. Overall Fault Detection Process

The pseudocode for the overall fault detection method based on dynamic LDA is as follows:

1. Each parameter of the normal historical samples *X*_0_ is normalized by *Z*-score to obtain ${\bar{X}}_{0}$
2. A sliding window with the length of *n*_1_ is used to extract the in-orbit data and *X*_*k*_ is obtained
3. The in-orbit data *X*_*k*_ is normalized by *Z*-score to obtain ${\bar{X}}_{k}$
4. LDA is used to find the optimal projection vector *w*_*k*_ between ${\bar{X}}_{0}$ and ${\bar{X}}_{k}$
5. A normal model is built using ${\bar{X}}_{0}$ and the optimal projection vector *w*_*k*_, and the detection threshold *ε*_*k*_ is obtained with the significance level *α*
6. The value of LDA objective function *J*(*w*_*k*_) is calculated according to equation (5)
7. Determine whether *J*(*w*_*k*_) is greater than 1/*n*_1_*ε*_*k*_ ?. If *J*(*w*_*k*_) > 1/*n*_1_*ε*_*k*_ was, the in-orbit data *X*_*k*_ is faulty; otherwise, *X*_*k*_ is normal. Let *k*=*k*+1, the in-orbit data *X*_*k*+1_ of next sliding window will be tested from Steps 3 to 7.

The computation cost of finding the optimum projection vector for each window mainly consists of matrix inversion, matrix multiplication, and solving eigenvalue problem. The time complexities of these three parts are *O*(*n*^3^), where *n* is the number of monitored variables. Considering all the aforementioned computation cost parts, the computation cost of finding the optimum projection vector for each window is *O*(*n*^3^).

## 4. Case Studies and Analysis

### 4.1. Numerical Case

#### 4.1.1. Experiment with the Fixed Fault Magnitude

A numerical simulation experiment which includes three faults was conducted to verify the effectiveness of the method proposed in this paper. The system was modeled as shown in

(18) $$\begin{array}{c} x_{1}=s_{1}+s_{2}+f_{1}+e_{1},\\ x_{2}=s_{1}-s_{3}+f_{1}+e_{2},\\ x_{3}=s_{1}-s_{4}+f_{1}+e_{3},\\ x_{4}=s_{2}+s_{3}+e_{4},\\ x_{5}=s_{2}-s_{4}+e_{5},\\ x_{6}=s_{2}+s_{4}+s_{5}+f_{2}+e_{6},\\ x_{7}=s_{3}-s_{4}+f_{3}+e_{7},\\ x_{8}=s_{3}-s_{5}+e_{8}. \end{array}$$

In equation (18), [*s*_1_, *s*_2_, *s*_3_, *s*_4_, *s*_5_]^*T*^ and [*e*_1_, *e*_2_, *e*_3_, *e*_4_, *e*_5_, *e*_6_, *e*_7_, *e*_8_]^*T*^ are independent Gaussian-distributed source signals and noises, respectively. All the source signals obey the standard normal distribution *ℕ*(0,1). *f*_1_, *f*_2_, and *f*_3_ are three incipient faults and do not occur simultaneously. *X*=[*x*_1_, *x*_2_, *x*_3_, *x*_4_, *x*_5_, *x*_6_, *x*_7_, *x*_8_]^*T*^ are the eight telemetry parameters that need to be monitored. All the fault types of *f*_1_, *f*_2_, and *f*_3_ are offset faults, as these faults occur more frequently in satellites. The three faults were inserted as shown in

(19) $$\begin{array}{c} f_{1}=\left\{\begin{array}{cc} 0 & 1\text{st}–30,100\text{th,}\\ 0.25 & 30,101\text{st}–60,200\text{th,} \end{array}\right.\\ f_{2}=\left\{\begin{array}{cc} 0 & 1\text{st}–30,100\text{th,}\\ 0.03 & 30,101\text{st}–60,200\text{th,} \end{array}\right.\\ f_{3}=\left\{\begin{array}{cc} 0 & 1\text{st}–30,100\text{th,}\\ 0.03 & 30,101\text{st}–60,200\text{th.} \end{array}\right. \end{array}$$

In this paper, four evaluation indexes: fault detection rate (FDR), false alarm rate (FAR), F1 value, and AUC value were chosen as the indexes for evaluating the fault detection results:

(20) $$\begin{array}{c} \text{FDR}=\text{prob}\left\{J\left(w_{k}\right)>\frac{1}{n_{1}\varepsilon_{k}}|H_{1}\right\}, \end{array}$$

(21) $$\begin{array}{c} \text{FAR}=\text{prob}\left\{J\left(w_{k}\right)>\frac{1}{n_{1}\varepsilon_{k}}|H_{0}\right\}, \end{array}$$

(22) $$\begin{array}{c} \text{FPR}=\text{prob}\left\{H_{1}|J\left(w_{k}\right)>\frac{1}{n_{1}\varepsilon_{k}}\right\}, \end{array}$$

(23) $$\begin{array}{c} F1=\frac{2*\text{FPR}*\text{FDR}}{\text{FPR}+\text{FDR}}. \end{array}$$

The other parameters of the numerical case were set as follows. The total number of samples was 120,400 of which 60,200 were normal historical samples and 60,200 were in-orbit samples for testing. The sliding window length was 300, and the sliding window interval was 100 for both the normal historical data and the in-orbit data in the experiment. After using sliding windows, both 600 windows were obtained from the normal historical data and the in-orbit data. The first 300 windows of the 600 windows of the in-orbit data were normal windows, while the last 300 windows were fault windows. The signal-to-noise ratio (SNR) was set to 30 dB [34].

In this paper, eight common fault detection methods were chosen as comparison methods, namely isolation forest (IForest) [35], OCSVM [36], *k*th nearest neighbor (KNN) [37], local outlier factor (LOF) [38], histogram-based outlier score (HBOS) [39], PCA with *T*^2^ statistic (PCA+*T*^2^) [19], PCA with squared prediction error statistic (PCA + SPE) [19], and PCA with combined index (PCA + CI) [40]. For comparison purposes, the parameters monitored by these eight methods were the mean values of each sliding window samples instead of the original values. IForest, OCSVM, KNN, LOF, and HBOS were implemented using the open-source program PyOD [41]. The parameters of PyOD are shown in Table 1. The significance of the parameters were detailed in Appendix (if there were no special explanations, other parameters were default values). For the three PCA-based fault detection methods, the cumulative variance contribution rate was 90%, and the confidence level of the statistic was set to 95%. The significance level of the proposed method was set to 0.005.

The detection results of nine fault detection methods for the fault *f*_1_ are shown in Figure 2. As can be seen from Figure 2, seven methods such as IForest, KNN, LOF, HBOS, PCA+*T*^2^, PCA + CI and the proposed method have satisfactory detection results for the fault *f*_1_, while the other two methods (OCSVM and PCA + SPE) have slightly poor detection results for the fault *f*_1_.

The detection results of nine fault detection methods for the fault *f*_2_ are shown in Figure 3. As is shown in Figure 3, the results of the first seven fault detection methods are not satisfactory for the fault *f*_2_. The fault or anomaly scores of these methods except OCSVM did not change significantly before and after insertion of the fault *f*_2_. Although the detection result of OCSVM is better, there are still a large number of fault windows below the threshold. It can be seen from Figure 3(i) that the proposed method has a good detection result for the fault *f*_2_.

As can be seen from Figure 4, except OCSVM and the proposed method, the other seven fault detection methods have poor performance in the detection of the fault *f*_3_. However, the detection result of OCSVM is not stable. In other words, due to randomly generated signal sources and noise sources, OCSVM may obtain good or poor results.

The three faults were simulated randomly 100 times in this paper [42], and then the average values of the fault detection results were calculated and are shown in Table 2.

As can be seen from Table 2, all the false alarm rate of the nine fault detection methods were concentrated in the vicinity of 5%∼7%. Consequently, it could be considered that the results in Table 2 are comparative results under similar false alarm rate condition. In terms of fault detection rate, the fault detection rate of the proposed method for the faults *f*_1_, *f*_2_, and *f*_3_ ranked 5th, 1st, and 1st, respectively. As for the fault *f*_1_, the proposed method ranked 5th but only 3.19% lower than the 1st method. In terms of F1 value, the F1 values of the proposed method for the faults *f*_1_, *f*_2_, and *f*_3_ ranked 5th, 1st, and 1st, respectively. In terms of AUC value, the AUC values of the proposed method for the faults *f*_1_, *f*_2_, and *f*_3_ ranked 3rd, 1st, and 1st, respectively.

Figure 5 shows the AUC value of 100 simulation results using OCSVM and proposed method to detect the fault *f*_3_. As can be seen from Figure 5, the detection results of OCSVM are unstable. Therefore, the evaluation index of OCSVM is not very high after averaging. On the contrary, the detection results of the proposed method are stable and satisfactory.

#### 4.1.2. Experiment with Different Fault Magnitudes

It is evident from Figure 4(i) that the proposed method has large allowances for the faults *f*_2_ and *f*_3_. In other words, it seems that the proposed method can also detect the smaller magnitude of the faults *f*_3_. To test the ability of detecting smaller faults of the proposed method, another experiment was conducted and the fault *f*_3_ was taken as an example. All the simulation environment and experimental parameters were retained, but the fault magnitude of *f*_3_ in equation (19) was varied. The fault magnitude of *f*_3_ was increased from 0.001 to 0.08, and the increase interval was 0.001. Each fault magnitude was simulated 30 times and the average value was used as the result. The F1 and AUC values of the detection results of nine methods with different fault magnitudes are shown in Figure 6.

As shown in Figures 6(a) and 6(b), the F1 and AUC values of the aforementioned nine methods show an increasing trend as the fault magnitude of *f*_3_ increases gradually, but the rate of increase varies among the nine methods. The F1 and AUC values of the proposed method increased rapidly with the increase of the fault magnitude and remained finally near the highest value. The optimal fault detection method of the other eight methods for the fault *f*_3_ was the OCSVM method, but it was slower than the method proposed in this paper. Due to the influence of noise, the detection result of OCSVM fluctuated greatly. As can be seen from Figure 6, the detection result of the proposed method may not be advantageous for large magnitude faults. However, in the case of incipient faults, the proposed method has an obvious advantage over the other eight fault detection methods. Therefore, the method proposed in this paper is more comprehensive in its ability to detect the different magnitudes of the fault *f*_3_.

#### 4.1.3. Analysis and Discussion

Why does the proposed method differ significantly in the detection of the faults *f*_1_, *f*_2_, and *f*_3_?. Why is the proposed method more sensitive to small-magnitude faults than other methods? This paper attempted to explain the reasons from the perspective of the optimal projection vector. For presentation purposes, the optimal projection vectors for each sliding window were normalized (the moduli of vector were set to 1) and taken the absolute value. The optimal projection vectors obtained by using dynamic LDA before and after the faults *f*_1_, *f*_2_, and *f*_3_ are shown in Figures 7(a)–7(c), respectively. In Figure 7, the first 300 windows were the normal windows, while the last 300 windows were the faulty windows.

As can be seen from Figure 7, due to the influence of noise, the optimal projection vectors obtained by the proposed method were chaotic and had no fixed pattern in the absence of faults. However, in Figures 7(b) and 7(c), the optimal projection vectors obtained using dynamic LDA showed regular patterns after faults *f*_2_ and *f*_3_ occurred. In comparison with Figure 7(a), the optimal projection vectors obtained using dynamic LDA were still chaotic after the occurrence of the fault *f*_1_, and there is no significant advantage between the proposed method and traditional methods:

(24) $$\begin{array}{c} w^{T}X=w_{1}x_{1}+w_{2}x_{2}+\cdots +w_{8}x_{8}. \end{array}$$

The size of each component of the optimal projection vector determines the degree of scaling of different parameters in *X*. Taking Figure 7(b) as an example, the weight of the parameter *x*_6_ was up to about 0.6 after the fault *f*_2_ occurred, while the weights of the parameters *x*_4_ and *x*_8_ were about 0.45, and the weights of the remaining parameters were below 0.3. It can be seen from equation (20) that the fault *f*_2_ was added to the parameter *x*_6_. It can be concluded that the optimal projection vector enlarged the weights of fault parameters and suppressed the weights of the other parameters. The enlargement of the fault parameters improves the ability of the proposed method to detect small-magnitude faults, while the suppression of the other parameters reduces the effect of noise from the other parameters.

As can be seen from Figure 7(c), the weights of *x*_3_ and *x*_7_ were significantly higher than the weights of the other parameters after the fault *f*_3_ occurred. It can be seen from equation (20) that the fault *f*_3_ was added to the parameter *x*_7_. It can be concluded that the optimal projection vectors also enlarged the weights of fault parameters and suppressed the weights of other parameters after the fault *f*_3_ occurred.

The traditional fault detection methods, such as OCSVM, IForest, and PCA, are static methods. Once the learning process is complete, they will use a fixed and invariable model to detect faults. Although the KNN method is dynamic, it treats each parameter equally. They did not have the aforementioned dynamic process of enlarging the weights of fault parameters and suppressing the weights of irrelevant parameters. Consequently, the other eight methods were not effective for the faults *f*_2_ and *f*_3_. Although OCSVM can obtain significant results sometimes, the detection results are not stable. After analysis, we consider that the instability of OCSVM may be caused by the selection of noise as the support vectors. In addition, comparing Figures 7(b) and 7(c), the optimal projection vectors were not the same for different faults. The optimal projection vectors obtained using the method proposed in this paper can be automatically adjusted according to the actual fault, and there is no need to manually set the parameter weights in advance.

### 4.2. Real Satellite Fault Case

On 28 June 2020, a fault occurred in a key component of a satellite payload. The postfailure analysis showed that the fault had been generated and developed over a long period of time. However, due to the first occurrence of the fault and the small magnitude of the initial failure, the fault was not detected and dealt with promptly. Finally, the status of the key component became unavailable. In this paper, a total of 1,315,515 samples of five telemetry parameters related to the faulty component were collected from satellite measurements and control systems from 12:15:04 on 10 November 2018 to 19:59:39 on 2 December 2019, as shown in Figure 8. For reasons of confidentiality, the true telemetry parameter names were hidden.

The first 266,540 samples of the total samples were selected as normal historical data, while the next 197,000 samples were selected as test data. The sliding window length was still set to 300 for both the test data and the normal historical data, but the sliding window interval was set to 100. After the sliding window extraction, a total of 2663 windows were obtained from the normal historical data, and a total of 1968 windows were obtained from the test data. The first 324 windows of the 1968 test windows were normal windows, while the subsequent windows were fault windows. The significance level of the proposed method was set to 0.0001, while the rest of the experimental parameters were the same as those presented in Section 4.1.1. The evaluation indexes and detection results of the nine fault detection methods for the real satellite fault are shown in Table 3 and Figure 9, respectively.

It can be summarized from Figure 9 that the four methods, which including OCSVM, KNN, LOF, and the proposed method, have better detection results for the real satellite fault. In terms of four evaluation indexes, the proposed method all obtained satisfactory results. Although the proposed method has little advantage over the other fault detection methods, it still ranked as the best that can be seen from Table 3. The effectiveness of the proposed method is further verified by the real satellite case.

## 5. Conclusions

Based on the analysis and comparison of existing satellite fault detection methods, this paper proposes a new incipient fault detection method that combines the core ideas of unsupervised learning and supervised learning. Then, the effectiveness and superiority of the proposed method were verified through a numerical simulation case and a real fault case. This paper only studies linear Gaussian system. If the system did not meet the assumptions of joint Gaussian distribution and linearity, the detection effect of the proposed method might decrease. Due to the insensitivity of LDA to variance, the proposed method is suitable for detecting the slight abnormal change of mean instead of the slight abnormal change of variance.

## Figures and Tables

**Figure 1:** Comparison of the uses of LDA: (a) traditional use of LDA and (b) the use of proposed LDA in this paper.

**Figure 2:** The detection results of five fault detection methods for the fault *f*_1_: (a) IForest result for *f*_1_, (b) OCSVM result for *f*_1_, (c) KNN result for *f*_1_, (d) LOF result for *f*_1_, (e) HBOS result for *f*_1_, (f)PCA+*T*^2^ result for *f*_1_, (g) PCA + SPE result for *f*_1_, (h) PCA + CI result for *f*_1_, and (i) the proposed method result for *f*_1_.

**Figure 3:** The detection results of five fault detection methods for the fault *f*_2_: (a) IForest result for *f*_2_, (b) OCSVM result for *f*_2_, (c) KNN result for *f*_2_, (d) LOF result for *f*_2_, (e) HBOS result for *f*_2_, (f)PCA+*T*^2^ result for *f*_2_, (g) PCA + SPE result for *f*_2_, (h) PCA + CI result for *f*_2_, and (i) the proposed method result for *f*_2_.

**Figure 4:** The detection results of five fault detection methods for the fault *f*_3_: (a) IForest result for *f*_3_, (b) OCSVM result for *f*_3_, (c) KNN result for *f*_3_, (d) LOF result for *f*_3_, (e) HBOS result for *f*_3_, (f)PCA+*T*^2^ result for *f*_3_, (g) PCA + SPE result for *f*_3_, (h) PCA + CI result for *f*_3_, and (i) the proposed method result for *f*_3_.

**Figure 5:** Detection results of two fault detection methods for the fault *f*_3_.

**Figure 6:** Comparison of fault detection results with different fault magnitudes: (a) F1 value for different fault magnitudes and (b) AUC value for different fault magnitudes.

**Figure 7:** Variation of optimal projection vectors for the different faults: (a) optimal projection vectors of *f*_1_, (b) optimal projection vectors of *f*_2_, and (c) optimal projection vectors of *f*_3_. From the perspective of projection, the projection process can be considered as a weighted sum process.

**Figure 8:** Raw telemetry data for fault-related parameters.

**Figure 9:** The detection results of five fault detection methods for the real satellite fault: (a) IForest method, (b) OCSVM method, (c) KNN method, (d) LOF method, (e) HBOS method, (f)PCA+*T*^2^ method, (g) PCA + SPE method, (h) PCA + CI method, and (i) the proposed method.

**Table 1:** Parameter settings of PyOD.

Method	Parameter settings
IForest	*n*_estimators = 100, contamination = 0.05
OCSVM	Kernel = ‘linear', nu = 0.6, contamination = 0.05
KNN	*n*_neighbors = 5, contamination = 0.05
LOF	*n*_neighbors = 20, contamination = 0.05
HBOS	*n*_bins = 10, alpha = 0.1, tol = 0.1, contamination = 0.05

**Table 2:** Comparison of fault detection performance for three faults.

Evaluation index	IForest	OCSVM	KNN	LOF	HBOS	PCA+*T*^2^	PCA + SPE	PCA + CI	Proposed method
FDR for *f*_1_ (%)	85.75	41.61	91.57	91.8	83.63	90.27	45.39	90.00	88.66
FAR for *f*_1_ (%)	5.37	5.31	6.07	6.49	5.96	5.68	5.61	5.64	4.95
F1 for *f*_1_	0.896	0.517	0.926	0.926	0.881	0.921	0.589	0.920	0.916
AUC for *f*_1_	0.964	0.791	0.977	0.976	0.957	0.978	0.804	0.978	0.976
FDR for *f*_2_ (%)	5.80	45.07	6.49	6.76	6.19	5.65	6.11	5.94	99.47
FAR for *f*_2_ (%)	5.37	5.13	5.85	6.34	5.71	5.10	5.87	5.75	4.86
F1 for *f*_2_	0.103	0.533	0.115	0.118	0.110	0.101	0.108	0.106	0.973
AUC for *f*_2_	0.511	0.794	0.522	0.516	0.509	0.507	0.537	0.517	0.998
FDR for *f*_3_ (%)	5.42	59.44	6.40	6.74	5.81	5.53	6.90	6.84	99.96
FAR for *f*_3_ (%)	5.48	5.37	5.92	6.14	5.79	5.40	5.70	5.54	5.07
F1 for *f*_3_	0.097	0.659	0.113	0.118	0.103	0.099	0.121	0.121	0.975
AUC for *f*_3_	0.506	0.856	0.522	0.514	0.503	0.500	0.560	0.523	1.000

**Table 3:** Comparison of fault detection performance for the real satellite fault.

Evaluation index	IForest	OCSVM	KNN	LOF	HBOS	PCA+*T*^2^	PCA + SPE	PCA + CI	Proposed method
FDR (%)	22.57	88.19	95.82	97.54	29.46	81.80	59.78	85.79	99.94
FAR (%)	2.05	7.60	9.65	12.28	2.63	3.22	2.34	1.75	1.17
F1	0.367	0.929	0.969	0.975	0.453	0.897	0.746	0.922	0.999
AUC	0.899	0.960	0.990	0.992	0.888	0.971	0.934	0.988	1

## Data Availability

The numerical case data used to support this study are included within the article. The real satellite fault data used to support the findings of this study are available from the corresponding author upon request.

## Appendix

The website of PyOD is https://github.com/yzhao062/Pyod.

  IForest *n*_estimators: the number of base estimators in the ensemble. contamination: the amount of contamination of the data set, that is, the proportion of outliers in the data set.
  OCSVM kernel: it specifies the kernel type to be used in the algorithm. nu: an upper bound on the fraction of training errors and a lower bound of the fraction of support vectors. contamination: the amount of contamination of the data set, i.e., the proportion of outliers in the data set.
  KNN *n*_neighbors: the number of neighbors to use by default for *k* neighbors queries. contamination: the amount of contamination of the data set, i.e., the proportion of outliers in the data set.
  LOF *n*_neighbors: the number of neighbors to use by default for *k* neighbors queries. contamination: the amount of contamination of the data set, i.e., the proportion of outliers in the data set.
  HBOS *n*_bins: the number of bins. alpha: the regularizer for preventing overflow. tol: the parameter to decide the flexibility while dealing the samples falling outside the bins. contamination: the amount of contamination of the data set, i.e., the proportion of outliers in the data set.
